RETRACTED

# Study on the Construction and Development Path of Gymnasiums considering Ecological Environment Restrictions

**DOI:** 10.1155/2022/2700957

**Published:** 2022-08-08

**Authors:** Xiaming Chen, Linhong Zheng, Yueyun Xu

**Affiliations:** ^1^Quanzhou Normal University, Quanzhou 362000, China; ^2^Centre for Sport and Exercise Sciences, University of Malaya, Kuala Lumpur 50603, Malaysia

## Abstract

Under the restriction of ecological and environmental factors, our requirements have improved for the development path of gymnasium construction. According to the previous way to carry out the development path of gymnasium construction will make our construction work encounter a lot of unnecessary troubles, so we can improve the success rate of the development path of gymnasium construction under the constraints of the ecological environment by carrying out relevant evasive operations according to the constraints of ecological environment. The topological path and path algorithm used to improve the efficiency of stadium construction and development path under the constraints of ecological environment, TEG algorithm, Q-TEG model, Q-TEG algorithm, Dtra algorithm, TraD algorithm, ResR algorithm, and Q-TED algorithm used in resource reservation plus time slot plus hosting bring the following advantages: (1) we use topological path and path algorithm to explore topological representation methods suitable for development path. The overview provides a theoretical basis for guidance, for forwarding technology scheduling mechanisms and multi-path forwarding mechanisms to provide higher flexibility. (2) We use the TEG algorithm of resource reservation plus time slot plus trusteeship, Q-TEG model, and Q-TEG algorithm under multi-model model can deal with the capacity and link of queue in each stadium construction development path well. It is more convenient to set the packet loss threshold for the propagation experiment tested in the simulation. Better help gymnasium construction and development path transmission is successful. (3) The use of the Dtra algorithm, TraD algorithm, ResR algorithm, and Q-TED algorithm in our stadium construction development path of a good deal of the transmission link structure between each node, so that the transmission efficiency between nodes becomes higher, making our stadium construction development path operation more efficient and convenient.

## 1. Introduction

The arid land in western China needs to be improved urgently, and the ecological environment in this arid area is of great significance to the implementation of national strategies and policies, the maintenance of social order, and the integration of land [1]. The research on ecological environment change, ecological environment degradation mechanism, and ecosystem regulation and control in the arid area can improve the structure and function of the ecosystem in spatial structure and ecosystem. There are signs of swamp degradation in Zoige Plateau, and the regional ecological environment and swamp ecosystem are seriously damaged, which is difficult to be restored by self-repair and artificial restoration. The deterioration of the ecological environment and swamp degradation cause the decrease of rare animal species and population, which provides the possibility for human activities to interfere [2]. The great decrease of phosphate concentration in Daya Bay leads to malnutrition level of seawater quality, and the seawater quality in the water system changes from nitrogen regulation to phosphorus regulation. The change of nutrient concentration in Daya Bay will lead to the miniaturization of the plant community [3]. Ecological fragility and agricultural activities jointly affect crop production in dry fields in the western Loess hilly and gully region. Effects of soil moisture and fertilizer content at different depths on slope and terrace ecology in Loess Plateau [4]. Muscle weakness and mechanical restriction can explain the decline of eyeball rotation and other common restrictions. The measurement of forced intraocular pressure difference and the study of saccade speed are helpful to record the existence of limitations. Limitation occurs after multiple ocular stiffness surgery caused by orbital floor fracture, orbital or retinal detachment surgery, and muscle displacement surgery [5]. A field experiment was conducted to study the soil nutrient restriction factors and plant nutrient absorption and accumulation of super-high-yield summer maize. The results showed that super-high-yielding summer maize could obtain better productivity under the influence of nutrient constraints; the growth period of super-high-yielding plants increased; and nutrient accumulation was the key period of nutrient absorption at the maximum maturity of the growth period [6]. Mass production of high-quality seeds, as a biological study of clonal seed orchards with obvious planning restrictions, can understand the flowering biology of oak trees with stems and produce high-quality seeds with high genetic diversity. Clones with different genotypes are helpful for pollination and ensure successful fertilization of seed quality and quantity. It is also important to synchronize the flowering and phenology of clones. The germination of oak stem buds is regulated by heredity, which provides the possibility for the correct selection of excellent trees [7]. E-government information resource sharing is the focus of national information system construction. At present, the main factors restricting the sharing of e-government information resources are insufficient information transmission, the low utilization rate of resources, and high cost of information sharing. Therefore, we should think about how to reform the means of information sharing services, strengthen the security management of information resource, and promote the development of e-government information resources sharing [8]. This section introduces some structures of Olympic venues. The structural schemes and corresponding construction technologies of these stadiums and gymnasium have genius thinking, which represents the discussion of the latest structural system of long-span spatial structures in China [9]. In order to ensure the high-quality completion of stadiums and gymnasiums construction and ensure the smooth holding of the national games, we can learn from the experience of stadiums and gymnasiums planning and construction in the past three national games through on-the-spot investigation and sorting out relevant documents at home and abroad. Based on the investigation of stadiums and gymnasiums in Shaanxi Province, the number, characteristics, overall layout, and construction methods of the required stadiums and gymnasiums are analyzed in detail, and then the functional orientation and construction standards of base facilities are put forward [10]. To provide scientific assessment and practical guidance for the construction and maintenance of sports lawns, mainly aiming at lawns that affect equipment maintenance in humid temperate climate. It describes general principles and has a section on identifying problems, components of drainage protection schemes, and functional implementation that can replace layout design guidelines [11]. The shortage of sports facilities in a region is reflected not only in the lack of key facilities but also in the rapid growth of the number of similar facilities. The conflict between the construction of community sports infrastructure and the development of community sports reflects the disadvantages of traditional construction. Infrastructure construction should not only rely on increasing investment but also coordinate sports facilities resources of enterprises and institutions and pay attention to system management and soft environment construction. Reasonable layout of infrastructure to meet the inherent requirements of sustainable development [12]. In recent years, the development path of electromagnetic energy conversion technology has made relevant breakthroughs. The utilization and recovery of these environmental electromagnetic energy is the most relevant and critical issue in the practical application of wireless energy acquisition equipment and systems at present and in the future. A simple measurement of the linear frequency of RF rectifier elements is successfully derived from emitter analysis [13]. The analysis of the development path in the economic sample reflects the value in the process of economic development. We use flexible path selection methods, in order to solve these possible contradictions, we have introduced a variety of nonparametric display models [14]. The research of biomaterials, the first generation of artificial bone substitute materials, established the concept of paving the way for commercialization. A new concept of amorphization is put forward so that the maximum compressive strength of hydrated materials is about 78 MPa [15].

RETRACTED

## 2. Related Narrations of Stadiums and Gymnasiums Construction under Ecological Environment

### 2.1. Problems in the Construction of Stadiums and Gymnasiums under Ecological Environment

The construction concept and development path of green venues based on ecological environment factors are starting, but at the same time, the destruction of the ecological environment is becoming more and more serious, resulting in very serious consequences. This situation brings great pressure to the development road of stadiums and gymnasiums in China. The negative impact of industrial development on the environment is unexpected. Although the economy has developed, it has sacrificed the environment, so serious ecological environment damage has appeared, which brings great resistance to the construction of stadiums and gymnasiums in China. Most data collection and analysis need to be based on real conditions, which poses a great challenge to the construction and development of our stadiums and gymnasiums. Because people's awareness of environmental protection has not been enhanced, it is difficult to walk out of a road of construction and development of stadiums and gymnasiums in an ecological environment.

### 2.2. Fundamental Guarantee for Stadium Construction and Development

The development path of stadiums and gymnasiums construction based on the ecological environment needs conditions and good ecological environment as the support of the big environment behind it. The significance of ecological environment protection construction is the fundamental guarantee for the development of social civilization because the progress and development of human society are the result of the common development of ecological, spiritual, material, and political civilization. Various civilizations blend, interact, and restrict each other. Doing all these well provides unique conditions for the construction and development of stadiums and gymnasiums in China. If we do a good job in ecological environment protection, we can rationally redistribute resources. Allocating better and more suitable resources for the construction and development of stadiums and gymnasiums and doing a good job in ecological environment protection are of great benefit to the construction of spiritual civilization. People's spiritual level has been improved, which is a green and healthy state for sports undertakings and sports construction.

RETRACTED

### 2.3. Establishing an Innovation Mechanism

It is necessary to have a new mechanism to facilitate the construction and development of stadiums and gymnasiums in the ecological environment. It is an important measure to establish an innovative mechanism of ecological environment protection. It is necessary to deeply study the needs of ecological environment protection in the new period and innovate environmental protection to establish good starting conditions and good development conditions for the construction and development of sports. First of all, the environmental protection department should become the connector between the government and enterprises. It is necessary to publicize the government's laws, regulations, and policies on environmental protection to enterprises. At the same time, we should report to the government the difficulties in environmental protection in the production and operation of enterprises and then find a balance between the government and enterprises so that relevant departments can join in as new forces and become new mechanisms and complete the innovative mechanism of ecological and environmental protection in the prevention stage so that the construction and development of our gymnasium will have more comparative advantages. A good mechanism can make the investment in gymnasium construction more effective and attract more capital. The accumulated investment in large-scale stadiums and gymnasiums in Fujian Province is 9.034 billion yuan, accounting for 30.72% of the investment in stadiums and gymnasiums in Fujian Province. Among them, the financial allocation is 5.828 billion yuan (only the sports charity fund allocates 426 million yuan, accounting for 7.32% of the government financial allocation), accounting for 64.51%. Self-raised funds are 2.753 billion yuan, accounting for 30.47%; social donations are 345 million yuan, accounting for 3.82%; and other investments are 10.91 billion yuan, accounting for 1.20%. Better mechanisms are conducive to investment in gymnasium construction.

## 3. Algorithm for the Development Path of Stadium Construction

### 3.1. Changes in the Development Path of Stadium Construction

When operating the development path of stadiums and gymnasiums, it meets the time certainty requirement of each sports construction path to the delay of subpaths. Generally, to achieve this goal, it is necessary to set the simulated relative coordinates according to the azimuth effect and optimize the relative position of the working path. One-to-one or one-to-many data transmission required for the construction and development channel of stadiums and gymnasiums is more convenient. In addition, because the gymnasium construction path can be backed up through multi-path transmission, the transmission location is often simplified to the description location. The relative position system divides the path space into grids and uses the grid method to represent the relative position. Based on the relative position, the following development path is constructed:

(1) $$\begin{array}{c} \left\{\begin{array}{c} X=\left(N+\text{alt}\right)\cos\left(\text{alt}\right)\cos\left(\text{lon}\right),\\ Y=\left(N+\text{alt}\right)\cos\left(\text{alt}\right)\sin\left(\text{lon}\right),\\ Z=\left(N\left(1-e^{2}\right)+\text{alt}\right)\sin\left(\text{lat}\right), \end{array}\right. \end{array}$$

where *e* is the offset rate of the reference relative position and *N* is the path value of the reference rate, and formula (1) is the decentralized calculation for calculating the path propagation of gymnasium construction. The relative coefficient of gymnasium construction is calculated with reference to the specific parameter value of gymnasium construction, and the specific calculation formula is as follows:

(2) $$\begin{array}{c} e^{2}=\frac{a^{2}-b^{2}}{a^{2}}, \end{array}$$

(3) $$\begin{array}{c} N=-\frac{a}{\sqrt{1-f\left(2-f\right)\sin^{2}\text{alt}}}. \end{array}$$

Because we need to arrange the path planning algorithm of the gymnasium before carrying out the development path of stadium construction, we also need to calculate the coordinates of relative positions on the grid map. If we can use coordinates to study the gymnasium construction path, it will greatly improve our resource utilization rate. It is more efficient to select the task area and specify the target for related operations according to the task needs.

RETRACTED

In the relative path construction of a gymnasium, there is a functional relationship between the extreme flattening rate *f*=(*a* − *b*)/*a*, the eccentricity distance *e*, and the extreme flattening rate *f*, and the maximum and minimum values of this functional relationship can be transformed by linear programming. Its specific expression formula is as follows:

(4) $$\begin{array}{c} e^{2}=f\left(2-f\right). \end{array}$$

In the development of the gymnasium path, it can be transformed by coordinates in the linear relationship formula. Among them, the coordinate transformation function formula of gymnasium construction can be expressed as follows:

(5) $$\begin{array}{c} \left\{\begin{array}{c} X=\left(N+\text{alt}\right)\cos\left(\text{lat}\right)\cos\left(\text{lon}\right),\\ Y=\left(N+\text{alt}\right)\cos\left(\text{lat}\right)\sin\left(\text{lon}\right),\\ Z=\left(N{\left(1-f\right)}^{2}+\text{alt}\right)\sin\left(\text{lat}\right). \end{array}\right. \end{array}$$

The relative position refers to the point *p* in radian, and the coordinates in UTM system are known values in km, which is in the development path of the gymnasium. You can set the position of the gymnasium to *p* first and then calculate the longitude zone where the *p* point is located. The calculation formula can be expressed as follows:

(6) $$\begin{array}{c} \text{Zonenum}=\left[\frac{\text{lon}}{6}\right]+1. \end{array}$$

The preparatory work we need to do before carrying out the development path of stadium construction, we need to sort out the nodes in the development path of the gymnasium, then allocate resources before transmission, determine the relative position, then reasonably allocate the data in the development path, then match the nodes, and then match the data after matching the nodes, and then, we need to set the location of the gymnasium for follow-up work.

*Z* is the longitude zone where the gymnasium is located. The relative inclination angle of the link area where the gymnasium is located is

(7) $$\begin{array}{c} {\text{lat}}_{0}=\left(\text{Zonenum}-1\right)*6-180+3. \end{array}$$

When we calculate the relative position of the stadium development path, we need to make clear the efficiency between each node and where the bearing range is, so as to achieve the optimization of resource allocation, the tasks within the specified time after the resource allocation, and the relevant standards set to measure the work efficiency of the conversion between nodes.

Then, the transformation intermediate variable of the relative path of the arena is calculated, which must be related to the relative coefficient in the relative linear programming function that determines the position of the relative path of the arena. Therefore, the specific functional relationship can be expressed as follows:

(8) $$\begin{array}{c} v\left(\text{lat}\right)=\frac{1}{\sqrt{1-e^{2}\sin^{2}\left(\text{lat}\right)}}. \end{array}$$

Before we carry out the stadium development path, we need to calculate the transformation intermediate variables of the stadium relative path. Then, we need to transform the data system of relative path, change it according to the correlation of relative coefficients in the relative linear programming function, and then reduce the system path of transforming intermediate variable data according to the appropriate situation.

RETRACTED

When calculating the relative path transformation of the gymnasium, the angle parameter must be considered. Angle parameters also have a function transformation relationship. The function of angle parameters and the function transformation relationship can be expressed as follows:

(9) $$\begin{array}{c} S\left(\text{lat}\right)=\left(1-\frac{e^{2}}{4}-\frac{3e^{2}}{64}-\frac{5e^{6}}{256}\right)\cdot \text{lat}-\left(\frac{3e^{2}}{8}+\frac{3e^{4}}{32}\right)\sin\left(2\text{lat}\right), \end{array}$$

(10) $$\begin{array}{c} c=\frac{e^{2}}{1-e^{2}}\cos^{2}\left(\text{lat}\right), \end{array}$$

(11) $$\begin{array}{c} E=E_{0}+k_{0}av\left(A+\left(1-T+C\right)\frac{A^{3}}{6}+\left(5-18T+T^{2}\right)\frac{A^{5}}{120}\right). \end{array}$$

Under environmental factors, our stadium construction and development path need to incorporate the angle parameters of specific reference objects. The change brought by the relative path change of the gymnasium will be a multi-angle change. According to the task needs, the task area should be selected, and then the central position should be analyzed to make a correct angle change choice, taking into account environmental factors and completing the construction path work at the same time.

The relative position of gymnasium construction and development path before transmission needs the path planning algorithm of the gymnasium to complete coordinate operation on a grid map, so it needs to be converted into UTM coordinates and then into map coordinate system. First, select the task area according to the task needs and then set one of the areas as the map origin; then the relative coordinates of any point are

(12) $$\begin{array}{c} N=N_{0}+k_{0}a\left(s+v\;\tan\;\varphi \left(\frac{A^{2}}{2}+\left(5-T+9C+4C^{2}\right)\frac{A^{4}}{24}\right)\right). \end{array}$$

Because the path planning algorithm of the gymnasium needs to calculate the relative position coordinates on the grid map, it is necessary to transform latitude and longitude coordinates into UTM coordinates and then transform them into map coordinates to study the gymnasium construction path. First, select the task area according to the task needs and set one of the areas as the map origin *p*, and the map coordinates of any point are

(13) $$\begin{array}{c} p_{E}^{\text{map}}=E-E_{\text{origin}}, \end{array}$$

(14) $$\begin{array}{c} p_{N}^{\text{map}}=E-E_{\text{origin}}. \end{array}$$

RETRACTED

### 3.2. Algorithm of Gymnasium Path Construction

A wheeled odometer is installed in the gymnasium. By observing the positions of the left and right sides, the relative path of the current gymnasium construction can be calculated. Because the gymnasium is a mobile building structure, the left and right positions are inconsistent and the positions are predicted. Considering the complexity of the predicted position model, the template model is used to replace it approximately. The angle value is expressed by the following formula, depending on the position of the template:

(15) $$\begin{array}{c} w=\frac{vr-vl}{2b}. \end{array}$$

In order to obtain a stable and continuous heading angle estimation of the relative path of the gymnasium, based on the filter of the position model of the gymnasium template, the system state vector is *x*=(*θ*, *ω*)^*T*^, and *w*=*θ*/*d*_*t*_ and *θ* can be observed, so the angular velocity calculated by the wheeled odometer is not observed, and only the angular velocity calculated by the wheeled odometer is used as the boundary constraint of the gymnasium engineering. The structural equation of the state of the system is as follows:

(16) $$\begin{array}{c} \left[\begin{array}{c} \theta_{k+1}\\ w_{k+1} \end{array}\right]=\left[\begin{array}{cc} J & △t\times U\\ 0 & I \end{array}\right]\left[\frac{\theta_{k}}{w_{k}}\right]+u, \end{array}$$

where *θ*_*k*+1_ and *w*_*k*+1_ are the route angle of *k*+1 frame and the angle of gymnasium project, respectively, and DD is the control quantity, which is set as the observation position because other sensors cannot measure it. The system state and covariance are first initialized when the first frame data arrives. The initialization expression is as follows:

(17) $$\begin{array}{c} \theta =\theta_{0},\\ w=0. \end{array}$$

We need to arrange the path planning algorithm of the gymnasium before carrying out the development path of stadium construction; there is good control of the route angle of the design framework and the angle of the gymnasium project. In order to calculate the relative system path relative to the gymnasium later, we need formula (17) to initialize the system state and covariance when the first frame data arrives. If it is missing, it will lead to slow path disorder.

(18) $$\begin{array}{c} {\mathrm{cov}}_{a}=\left[\begin{array}{cc} 0.2 & 0\\ 0 & 0.2 \end{array}\right]. \end{array}$$

According to the gymnasium construction model, the relative system path relative to the gymnasium can be calculated, and the relative path changes with time. Therefore, in order to study the relative path of the gymnasium, it is necessary to calculate the predicted value of the system state at the next moment. The calculation method of the predicted value is as follows:

(19) $$\begin{array}{c} \theta_{k+1}=\theta_{k}+wt, \end{array}$$

(20) $$\begin{array}{c} w_{k+1}=wk. \end{array}$$

The angle calculation of the gymnasium construction road path has true value and predicted value. We introduce covariance to predict the angle of the gymnasium path, so as to accurately estimate the angle between the true value and the gymnasium path. The covariance prediction value at the next time is as follows:

(21) $$\begin{array}{c} {\mathrm{cov}}_{\text{pre}}=F{\mathrm{cov}}_{k}F^{T}, \end{array}$$

where *F* is the position matrix of state transition gymnasium construction and *d*_*t*_ is the position spacing between two measurements, and the specific formula is

(22) $$\begin{array}{c} F=\left[\begin{array}{cc} I & d_{t}\\ 0 & I \end{array}\right]. \end{array}$$

Waiting for the arrival of the next frame of data, the difference error between the previous gymnasium model route angle prediction value *θ*_pre_ and the actual gymnasium construction route angle observation value *θ*_abs_ is calculated, and finally, the best position estimation value and the worst predicted construction position estimation value are calculated. The best state estimation is as follows:

(23) $$\begin{array}{c} \text{error}=\theta_{\text{obs}}-\theta_{\text{pre}}. \end{array}$$

The best position estimate and the best error estimate are calculated. The best position estimation needs to be verified after obtaining the best position model of *K*+1 frame. Because the construction of the gymnasium needs to meet the proper planning, the pitch angle difference of *K*+1 frame is not greater than Δ*θ*_max_, that is, max is the maximum pitch angle difference between the two frames. The heading angle expression can be expressed as follows:

(24) $$\begin{array}{c} |\theta_{k+1}-\theta_{k}|\leq \Delta \theta_{\max}, \end{array}$$

where *w*_max_ is the maximum heading angle difference between two frames and *d*_*t*_ is the position interval between two frames. The data output frequency of the positioning system used in this paper is about 20 Hz, so *d*_*t*_ is used. The specific calculation method is as follows:

(25) $$\begin{array}{c} w_{\max}=\min\left[w_{\text{atr}},w_{\text{odom}}\right]. \end{array}$$

In formula (25), according to the observation of the construction data of the left and right wheel positions of the wheel odometer, the construction position angle of specific facilities in the gymnasium and the best construction position that the gymnasium construction model can achieve are calculated. Locations are selected from the actual model built around the gymnasium. Black dots represent positions, and the multi-segment lines connecting positions do not match the actual positions. The placement satisfies the multi-path position constraint, and the system path position expression is as follows:

(26) $$\begin{array}{c} \left[\begin{array}{c} x_{k+1}\\ v_{k+1} \end{array}\right]=\left[\begin{array}{cc} I & \Delta t\times I\\ 0 & I \end{array}\right]\left[\begin{array}{c} x_{k}\\ v_{k} \end{array}\right]+u. \end{array}$$

RETRACTED

## 4. Related Operations of Gymnasium Construction and Development Path

### 4.1. Comparative Analysis of the Construction and Operation Modes of Stadiums and Gymnasiums

The operation modes of stadiums and gymnasiums include but are not limited to independent operation, cooperative operation, and entrusted operation. Due to different resources and constraints, each operation mode has its own characteristics and limitations, but the goal is the same. All these can promote the management efficiency of stadiums and gymnasiums on the premise of ensuring social benefits, thus improving economic benefits. According to the census data, 93.7% of large stadiums and gymnasiums in Fujian Province adopt independent operation mode; 4.5% adopt entrusted operation mode; and only 1.8% adopt cooperative operation mode. It is found that Pearson Kay Square is 31.098a, *P*=0.000 < 0.05, indicating that there is a significant correlation between the operation modes and types of large stadiums in Fujian Province. The absolute values of residual value adjustment of stadiums, swimming venues, and operation modes are 4.1, 2.1, 3.5, 5.4, 3.4, and 4.2, respectively, and they are not less than 1.96, indicating that the number of independent operations of stadiums and gymnasiums in Fujian Province is obviously higher than that of independent operation, and the proportion of cooperative operation and entrusted operation of swimming venues is more than that of cooperative operation and entrusted operation of stadiums and gymnasiums. However, there is no significant correlation between gymnasium and operation mode (the adjustment numbers of residual value are 1.2, 1.48, and 0.5, respectively, which are less than 1.96). Although there are differences in the operation modes of stadiums and gymnasiums in Fujian, on the whole, the ownership and operation rights of most stadiums and gymnasiums in Fujian are consistent. Sports venues and markets are not well integrated. In addition, the division of labor level is low, and the management concept and means are relatively lagging behind. Due to the excessive protection of the administrative system, the market lacks competitiveness. Among them, the gym performed well and the swimming pool performed relatively well. The operation modes and types of large stadiums and gymnasiums in Fujian Province are shown in Table 1.

RETRACTED

These large stadiums and gymnasiums undertake various cultural and sports activities, and these subjects also suffer losses due to the increase in maintenance costs. In recent years, the state regulates the operation of stadiums and gymnasiums, but their profitability has not been strong. According to the census data, the proportion of loss-making stadiums and gymnasiums is 6.77%; the proportion of profit-making stadiums and gymnasiums is 23.3%; and the proportion of flat-operating stadiums and gymnasiums is 70.0%. Some venues lost 6.1 million yuan, while others brought in more than 1 million yuan in income a year. Chi-square test of a contingency table is used to test the management effect and operation effect of large stadiums and gymnasiums: Pearson's chi-square is 20.774a, *P*=0.000 < 0.05, which shows that the management mode of large stadiums and gymnasiums in Fujian Province is significantly related to the management situation. The absolute values of surplus, balance, and operation mode adjustment surplus are 4.4, 2.7, 3.4, 4.1, 2.0, and 3.5, respectively, indicating that the number of cooperative operation and entrusted operation of surplus-scale stadiums is significantly higher than that of independent operation, and the proportion of independent operation of flat-scale stadiums is significantly higher than that of cooperative operation and entrusted operation. However, there is no obvious difference between venues with loss scale and operation mode (the absolute value of adjusted surplus is 0.0, 0.8, and 0.6 < 1.96), which shows that the profit and loss of large venues are closely related to operation, management authority distribution, and asset structure. See Table 2 for the operation mode and profit rate of large venues in Fujian Province:

With the steady development of China's social economy and the continuous improvement of people's demand for sports, Fujian makes full use of its location advantages to carrying out colorful sports activities. According to the census data, there are 2,381 employees in 443 stadiums and gymnasiums in Fujian Province, with a total opening hour of 76,998 days. The income of large and small stadiums and gymnasiums includes financial allocation, extra budgetary funds of administrative units, subsidy income of higher authorities, business income of public institutions, income turned over by subordinate units and other income, and operating income and nonoperating income of stadiums and gymnasiums. The total investment in the project is 597.014 million yuan. The expenses paid by sports facilities of all scales (including supporting houses) totaled 585.799 million yuan, and the total profit was 11.215 million yuan. Among them, the number of employees and annual opening days of swimming pools ranks first, while the stadium has the highest total revenue and expenditure due to its large scale. From the perspective of single-scale stadiums and gymnasiums, the average number of employees in single-scale stadiums and gymnasiums in Fujian Province is 5, one less than the national average. The average annual open day is 174 days, which is 7 days more than the national average; the per capita income is 1.348 million yuan, which is 765,000 yuan higher than the national average; and the average expenditure on educational facilities is 132,200 yuan, which is 734,000 yuan higher than the national average. Among them, the average annual income of employees is 251,000 yuan, which is 153,000 yuan higher than the national average; the average profit is 5,000 yuan, which is 6,000 yuan higher than the national average. It can be seen that the operating cost of large stadiums in Fujian Province is higher than the national average. They generally bring benefits, but due to the low-performance index, the profitability is often limited, as shown in Table 3.

RETRACTED

### 4.2. Deterministic Technical Analysis of the Development Path of Gymnasium Construction

The construction of large-scale stadiums and gymnasiums is going on. In order to put forward a constructive solution for the transmission of stadiums and gymnasiums development path, the processing of the secondary path construction path of each stadium and gymnasium can effectively reduce the packet loss in the construction path and ensure the reliability of the construction path while ensuring the certainty of transmission. Therefore, this paper mainly explores the deterministic multi-path-related technology of gymnasium path construction from two aspects: related protocols and path transmission. Transmission protocol provides multiple transmission paths with delay guarantee for deterministic multi-path transmission, and path transmission guarantee provides accurate multi-path scheme according to construction requirements and carries out the deterministic transmission on construction paths. Explore the path technology of gymnasium construction, This paper mainly summarizes the clear transmission and display methods of sports construction development path from two aspects of topological path and path algorithm, This paper summarizes the existing multi-path algorithms, which provides theoretical guidance for the construction of the transmission multi-path algorithm of the development path of sports construction, and provides a reference for the design of packet scheduling mechanism and multi-path transmission protocol.  Figure 1 shows its contents:

The traditional path uses the transmission resources of the gymnasium path to reserve time slots. Under the scheduling strategy of resource reservation + time slot + managed TEG algorithm, path packet loss often occurs in the transmission process. The performance of various transmission strategies of gymnasium construction paths is compared, which ensures the reliability of data packets. TEC experiment simulates data packets with less time period and generates uniformly distributed arbitrary paths, which can meet the requirements of service delay. The link width of the simulation path is 50 Gbps, and the length of the time slot is 8 ms. After the TEG model is established, the sending queue data of the managed gymnasium path is set to 8, and the data packets generated successively are numbered and sent, simulating the sending process of the data packets in each node and recording the data points where the data packets sent by each gymnasium arrive at each node. When a packet arrives at the same node at the same time, it is regarded as packet loss. According to this, the reliability and guarantee performance of various transmission strategies for sports engineering path data packet transmission under different network loads are counted. The transmission error rate by scheduling condition is shown in Figure 2.

RETRACTED

Because before scheduling the resources in the development path of sports construction, we must first make a concrete analysis of reserving time slots for transmission resources. In order to reduce the occurrence of packet loss and improve the performance of the gymnasium construction path transmission strategy, the link width of the simulation path is not the same, and the quality and size of the data sent in the queue are also different under different network loads, so the gap may be obvious.

Considering the ecological environment constraints, we set different QS parameters, which restrict the success rate of the Q-TEG algorithm in selecting and arranging the development path of sports construction. This simulation experiment explores the influence of different QS parameters on the performance of the Q-TEG algorithm. For each link of the shown gymnasium building path topology, a small random error rate is set in addition to the basic path propagation delay bandwidth parameter. The propagation parameters of the development path of sports construction are fixed values, which are calculated according to distance. The Q-TEG model is constructed with the time slot length *t* = 8 ms, the number of node queues needs to be recorded, and the capacity of each queue matches the capacity of links when the propagation movement constructs the development path. According to the propagation experiment of the simulation test, the packet loss threshold is randomly set at the beginning node and the end node of the development path of gymnasium construction. Whether the development path transmission of gymnasium construction is successful and whether the upper limit of delay, the upper limit of path jitter, the upper limit of loss of inclusion, and service arrangement are successful, the transmission compliance rate of development paths in different directions is shown in Figure 3.

RETRACTED

### 4.3. Breakthrough of Restrictive Factors in the Path of Sports Development and Construction

From the above simulation results, it can be seen that the Q-TEG algorithm, compared with the traditional Dtra algorithm and the Dtra algorithm supporting resource reservation, has certain limitations on the scheduling completion rate of gymnasium construction path development. The link bandwidth of the sports construction development path has a great influence on transmission, and sports construction development has a great influence on the completion rate through single- or multi-channel scheduling. Under the condition of sufficient link bandwidth, due to time constraints, fluctuation constraints, and packet loss constraints, the propagation layout of the sports construction development path cannot be completed. Packet loss rate rarely occurs in multi-path, which proves that multi-path is more efficient in controlling the development path of sports construction and controls packet loss in a very small range. Because the jitter of any path of Q-TEG is fixed at 2 in different variation intervals, when the variation threshold is relaxed, the varying path time difference and path intrinsically become relaxed for a single path to multi-path. The slot length of the Q-TEG model and the multi-path delay difference of the Q-TEG model in multi-path configuration can bring better performance to the algorithm. The comparison of sports construction development paths under different change thresholds is shown in Figure 4.

The propagation parameters of the path are fixed when the development path of stadium construction is carried out, and the capacity of the queue matches the capacity of the link when the propagation movement constructs the development path so that the ecological environment constraints can be taken into account and the random error rate of the path can be reduced. Multi-path has higher controllable efficiency for the development path of sports construction, and the performance of the derived protection mechanism and single-route retransmission guarantee mechanism is also guaranteed, which is more conducive to the work.

RETRACTED

In order to break through the limitation of timeliness, this paper compares the performance of multi-path sports construction routing service protection mechanism and single-route retransmission guarantee mechanism in timeliness deterministic transmission network and analyzes the performance of the two mechanisms in effective timeliness. The invalid transmission rate of data packets refers to the ratio of the lost data packets and the total number of transmitted data packets in the transmission process of the sports construction development path. In order to prevent packet loss, it is necessary to analyze the formation of problems and constraints. However, we believe that the lower the packet loss rate, the better. We compare the transmission efficiency and constraint breakthrough probability under different algorithms, as shown in Table 4.

In the process of developing a mobile engineering path, the original data of path vertices without path base points in these single paths are processed and deleted, and the shortest path index with other vertices is made for each vertex with remaining simplified data. Before constructing the processing strategy, calculate the priority of each vertex in the development path of sports construction, take the priority of vertex as the processing order of index construction, and query the constructed index at the same time of index construction. If the result of searching for the shortest path of an update object vertex from the constructed index is greater than the shortest path index of the constructed object, the index of the update object vertex is ignored. When the shortest path index is smaller than the shortest path index that should be constructed among the constructed shortest path indexes, the shortest path index of the updated vertex is maintained. Retrieval association constraints depend on the development path data constructed by the index. Comparative analysis of the construction effects of transmission on different paths can be seen in Table 5.

### 4.4. Strengthening the Path of Construction and Development under Environmental Factors

The method of strengthening the development path of venue construction requires establishing a model according to the environmental impact, considering the relationship with environmental factors when facing complex problems, and calculating, storing, and reusing the solutions of each subproblem. In consideration of environmental factors on the basis of current situation analysis, first initialize the path data of gymnasium construction, convenient for later path analysis. The optimal strategy is adopted to enhance the transmission state of the simulation path and make it interact with the environment all the time. After deciding to implement, according to the implementation effect, analyze how to optimize the governance under environmental factors and finally achieve the goal. The current construction work needs to collect or build data in advance and set the development path under environmental factors according to the existing static data. Enhanced path data generation and model optimization are combined in an interactive way, and the optimization process is fed back to the network model for repeated optimization processing, so it is suitable for the early planning of gymnasium construction path development. In the preliminary analysis, combined with the influence of environmental factors, the following work can be done, as shown in Figure 5.

RETRACTED

In the process of optimizing the development path of gymnasium construction, we need to feedback on the network model and carry out repeated optimization processing, The later path analysis needs to be established within the fluctuation range of the simulation path, which is convenient for the subsequent interactive operation of the environment. Analyze the environmental factors and set the development path under the environmental factors according to the existing static data and then choose the suitable preplanning of the gymnasium construction path development.

Through the above combined with the current environmental factors to deal with the development path, we found the best path for the initial node and the end node of the development path in the process of gymnasium construction. Because nonoverlapping paths between nodes must be calculated, paths cannot contain loops, and there cannot be overlapping nodes between different paths. Different algorithms are used to analyze and compare the operations under different path intervals. After each search, the nodes on the path will be isolated. Cut off all edges of nodes on the path, transform them into isolated nodes, and generate a new network graph. This is the number of nonrepeated paths between nodes. Using the concept of optimal path and node separation in the search process can ensure the actual requirements of paths and make up for the shortcomings of repeated path nodes.  Figure 6 below shows the behavior comparison:

When the path processing effect used in the stadium development path is not good, We need to find out the number of nonrepeated paths between nodes and then deal with the development path according to the current environmental factors, cut off all edges of nodes on the path, isolate unavailable nodes, and finally ensure the actual requirements of the path.

RETRACTED

Considering the time consumption of path numbers caused by environmental factors, the time consumption of the nonrepeated path algorithm and BFS technique is adopted. Based on the matrix power path algorithm and acyclic path algorithm, the development mode of gymnasium construction under the influence of environmental factors is optimized, considering that the required time is similar to the above. Based on the principle of the optimization method, this paper analyzes the limitation of environmental factors on the development path of gymnasium construction. Considering that in the process of calculating the path without a loop, the intermediate matrix is obtained by multiplying the number of paths in the previous layer with the adjacent matrix every time and then new expansion nodes are added to lead to the circular path, the corresponding number is eliminated from the intermediate matrix. The results of analyzing the power of the matrix show that the number of paths between nodes in the network can be obtained from the K power of the matrix. In the calculation of the number of paths, because both algorithms use a large number of matrix multiplication operations, there is a similar time. The acyclic path is based on the power of the matrix, plus the acyclic operation, so the final result is more accurate than the power multiplication of the matrix. The width-first search method takes the most time. According to the method analysis, after determining one path, delete the corresponding build path node. The width-first search method takes the longest time because it requires repeated searches in the network. In this algorithm, based on the starting point node and the end point node of the path, the best path is selected as the subpath for connection. Multiple iterations are avoided when finding nodes. According to the limitations of different environmental factors, the efficiency comparison results of the selected methods on the path are shown in Figure 7.

Compared with the traditional treatment of gymnasium construction and development path under environmental factors, it is necessary to clearly understand the number of nonrepetitive path calculations. It can be seen that with the increase of node scale based on the construction path, we need to deal with the analysis data received in real time under environmental constraints, and the calculation results will improve the effect of the gymnasium construction and development path more obviously. The recirculation path elimination algorithm is based on a matrix path, which eliminates most of the number of recycling paths but includes the number of repeated nodes between paths, and the calculation result becomes larger. The algorithm explores the development path of gymnasium construction and considers the actual needs. When there are multiple paths between nodes, there are many cases of choosing the best path. The key nodes are selected from the cross set of the starting node and the end node, and the path splicing method is used to calculate the nonrepeating path. The result is more accurate than the path power method, reducing most cyclic paths and iterative paths of some nodes. The current node has connected candidate nodes, and the repeated paths are found by the width-first algorithm, and the elimination efficiency of repeated paths in different path intervals is compared, as shown in Figure 8.

RETRACTED

## 5. Concluding Remarks

This paper deeply analyzes the treatment methods of the development path of gymnasium construction under the restriction of environmental factors that should be faced: what problems should we take into account in order to better improve the transmission efficiency of gymnasium construction and development path under the restriction of environmental factors, how to break through the limitations of environmental factors, and how to operate the development path more efficiently. We mainly develop the characterization method from two aspects: topological path and path algorithm. Explore the multi-path algorithm of deterministic development path to carry out the related operation of preliminary gymnasium construction development path. We also use the Q-TEG algorithm under multiple models to arrange the development of gymnasium construction path with high completion rate. Compared with the traditional Dtra algorithm, it is convenient for us to make transmission strategies and improve the performance of data packet reliability guarantee. Operationally, it provides us with great support for the development path of gymnasium construction under the influence of environmental factors. The comprehensive use of these methods and set models also makes us more effective in data utilization and more comprehensive protection in the transmission process of gymnasium construction development path transmission.

## Figures and Tables

**Figure 1:** Communication operation of gymnasium construction and development path.

**Figure 2:** Comparison of error rates under different scheduling conditions.

**Figure 3:** Completion rate of gymnasium construction and development path in different directions.

**Figure 4:** Breakthrough completion of sports construction development path under different fluctuation thresholds.

RETRACTED

**Figure 5:** Strengthening process of stadium construction and development path.

**Figure 6:** Comparison of optimization effects of different algorithm development paths.

**Figure 7:** Efficiency comparison results of path methods.

**Figure 8:** Comparison of algorithm repeated path elimination efficiency in different path segments.

**Table 1:** Operation modes and types of large-scale stadiums in Fujian Province.

Type		Independent operation	Cooperative operation	Entrusted operation	Total
Scale stadium	Total	212	1	2	215
	Percentage	51.1%	12.5%	10.0%	48.5%
	Adjustment of residual value	4.1	−2.1	−3.5	

Gymnasium	Total	83	0	3	86
	Percentage	20.0%	0.0%	15.0%	19.4%
	Adjustment of residual value	1.2	−1.4	−0.5	

Natatorium	Total	120	7	15	142
	Percentage	28.9%	87.5%	75.0%	32.1%
	Adjustment of residual value	−5.4	3.4	4.2	

Total	Total	415	8	20	443
	Percentage	100.0%	100.0%	100.0%	100.0%

**Table 2:** Operation mode and profit rate of scale sports venues in Fujian province.

Type		Profit	Balance	Deficit	Total
Independent operation	Total	87	300	28	415
	Percentage	84.5%	96.8%	93.3%	93.7%
	Adjustment of residual value	−4.4	4.1	0.0	

Cooperative operation	Total	5	3	0	8
	Percentage	4.9%	1.0%	0.0%	1.8%
	Adjustment of residual value	2.7	−2.0	−0.8	

Entrusted cooperation	Total	11	7	2	20
	Percentage	10.7%	2.3%	6.7%	4.5%
	Adjustment of residual value	3.4	−3.5	0.6	

Total	Total	103	310	30	443
	Percentage	100.0%	100.0%	100.0%	100.0%

**Table 3:** The operation comparison between Fujian and China.

Type		Employees		Opening days in a year		Total income (thousand yuan)		Total expenditure (thousand yuan)	
Fujian	Sports ground	541	3	34,746	162	460,312	2,141	458,581	2,133
	Stadium	439	5	13,028	151	36,680	427	39,168	455
	Natatorium	1,401	10	29,224	206	100,022	704	88,050	620
	Diving hall	0	0	0	0	0	0	0	0
	Total	2381	5	76,998	174	597,014	1,348	585,799	1,322

China	Sports ground	18,950	3	780,541	138	2,160,965	381	2,081,736	367
	Stadium	18,853	6	528,101	173	2,010,931	658	2,586,091	847
	Natatorium	32,937	10	672,477	212	2,705,021	855	2,266,820	716
	Diving hall	336	11	3,043	101	68,884	2,296	69,024	2,301
	Total	71,076	6	1,984,162	167	6,945,801	583	7,003,671	588

**Table 4:** The transmission efficiency and the probability of breaking through the limiting factors under different algorithms are compared.

	Propagation efficiency of single path	Multipath propagation efficiency	Limiting factor resolution rate
Dtra	0.845	0.356	0.18
ResR	0.956	0.548	0.26
Q-TED	0.984	0.628	0.34

**Table 5:** Comparative analysis of index propagation effect on different paths.

Index set	PLL	IS-ABLE	SHP	CP
Xmark	109	151	121	121
Vchocyc	221	278	198	187
Amaze	56	89	78	84
Anthra	241	324	256	202

## Data Availability

The experimental data used to support the findings of this study are available from the corresponding author upon request.
